The article "Osteogenic protein-1 alleviates high glucose microenvironment-caused degenerative changes in nucleus pulposus cells" was retracted in 2024. Reasons: duplicated images; concerns about the peer review; concerns about the authorship.

# Osteogenic protein-1 alleviates high glucose microenvironment-caused degenerative changes in nucleus pulposus cells

**DOI:** 10.1042/BSR20190170

**Published:** 2019-04-02

**Authors:** Ziming Liu, Zhiwen Zhang, Ali Zhang, Fan Zhang, Wennan Du, Yongqiang Zhang, Rongfeng Zhang, Jiagang Xu, Xiangkun Wu, Chengmin Zhang, Ning Li, Qi Tan, Wei Huang

**Affiliations:** 1 Department of Joint Surgery, First Affiliated Hospital of Chongqing Medical University, Chongqing, China; 2 Department of Traditional Chinese Traumatology, Hubei Provincial Hospital of Traditional Chinese Medicine, Wuhan, Hubei, 430061, China; Department of Traditional Chinese Traumatology, Hubei Province Academy of Traditional Chinese Medicine, Wuhan, Hubei 430070, China; 3 Department of Orthopedic Surgery, The 80th Army Hospital of People’s Liberation Army (no. 89 Hospital of People’s Liberation Army), Weifang 261025, Shandong, China; 4 Department of Pharmacy, The 80th Army Hospital of People’s Liberation Army (no. 89 Hospital of People’s Liberation Army), Weifang 261025, Shandong, China; 5 Department of Medical Service, The 80th Army Hospital of People’s Liberation Army (no. 89 Hospital of People’s Liberation Army), Weifang 261025, Shandong, China; 6 Department of Orthopedic Surgery, Southwest Hospital, Third Military Medical University, Chongqing, China; 7 Nursing Department, Weifang People’s Hospital, Weifang, Shandong, China

**Keywords:** apoptosis, high glucose, intervertebral disc degeneration, nucleus pulposus, osteogenic protein-1

## Abstract

Increasing evidence has indicated a close relationship between diabetes mellitus (DM) and disc degeneration. As a potential therapeutic growth factor, osteogenic protein-1 (OP-1) has lots of protective effects on the healthy disc cell’s biology. The present study was aimed to investigate the effects of OP-1 on degenerative changes of nucleus pulposus (NP) cells in a high glucose culture. Rat NP cells were cultured in the baseline medium or the high glucose (0.2 M) culture medium. OP-1 was added into the high glucose culture medium to investigate whether its has some protective effects against degenerative changes of NP cells in the high glucose culture. NP cell apoptosis ratio, caspase-3/9 activity, expression of apoptosis-related molecules (Bcl-2, Bax, and caspase-3), matrix macromolecules (aggrecan and collagen II), and matrix remodeling enzymes (MMP-3, MMP-13, and ADAMTS-4), and immuno-staining of NP matrix proteins (aggrecan and collagen II) were evaluated. Compared with the baseline culture, high glucose culture significantly increased NP cell apoptosis ratio, caspase-3/9 activity, up-regulated expression of Bax, caspase-3, MMP-3, MMP-13 and ADAMTS-4, down-regulated expression of Bcl-2, aggrecan and collagen II, and decreased staining intensity of aggrecan and collagen II. However, the results of these parameters were partly reversed by the addition of OP-1 in the high glucose culture. OP-1 can alleviate high glucose microenvironment-induced degenerative changes of NP cells. The present study provides that OP-1 may be promising in retarding disc degeneration in DM patients.

## Introduction

Low back pain is a common musculoskeletal disease around the world. Intervertebral disc degeneration, occurring in ∼40% of these cases, is regarded as a main contributor to low back pain [1]. Currently, the number of patients with intervertebral disc degeneration is increasing due to the population ageing in the world, which causes lots of medical spending [2]. Though large amount of research projects are authorized to explore the mechanisms of disc degeneration [3–8], the pathogenesis is still not clear to us and no effective prevent strategy is developed to retard disc degeneration.

Increasing evidence has indicated that diabetes mellitus (DM) is a potential etiological factor of disc degeneration [9–12]. Hyperglycemia is a major reason of diabetes-related complications. Previous studies have shown that glucose-mediated oxidative stress injury is associated with hyperglycemia [13,14]. Importantly, oxidative stress injury caused by the increase in intracellular reactive oxygen species (ROS) seriously and negatively affects disc cell biology [3,15–17]. Moreover, high glucose microenvironment has been proved to promote degenerative changes in disc cells [9,11,18–23]. Therefore, inhibition of high glucose environment-induced harmful effects may be important in retarding disc degeneration in DM patients.

Osteogenic protein-1 (OP-1) is reported to stimulate disc matrix anabolism and protect healthy disc cell’s biology *in vivo* and *in vitro* [24–28]. However, whether OP-1 is effective in inhibiting high glucose environment-induced degenerative changes of disc nucleus pulposus (NP) cells remains unclear. Hence, the present study is aimed to investigate the effects of OP-1 on the degenerative changes of NP cells in a high glucose microenvironment. Some parameters, such as cell apoptosis, NP matrix protein synthesis, and expression of matrix remodeling enzymes, were investigated.

## Materials and methods

### Ethical statement

A total of 34 Sprague-Dawley rats were used according to guideline of the Ethics Committee at the First Affiliated Hospital of Chongqing Medical University.

### NP cell isolation and culture

After experimental animals were killed, the individual discs (T11-L5) were separated and put into a 50-ml centrifuge tube containing sterile phosphate buffer solution (PBS). Then, the central NP tissue was isolated using a medicine spoon and cut into small pieces (1 × 1 × 1 mm). After the isolated NP tissues were digested by 0.02% collagenase (Sigma-Aldrich, U.S.A.) overnight at 37°C, NP cell pellets were obtained by centrifugation and resuspended in DMEM/F12 culture medium. NP cells were cultured in baseline DMEM/F12 medium containing 10% fetal bovine serum (FBS, Gibco, U.S.A.) without a high glucose concentration (0.2 M, control group) or with a high glucose concentration (0.2 M, experiment group) for 10 days in a CO_2_ incubator (37°C, 21% O_2_, and 5% CO_2_). OP-1 (100 ng/ml) was added along with the culture medium with a high glucose concentration to investigate its protective effects. The concentration of OP-1 is determined according to a previous study [29].

### Flow cytometry analysis

After culture, NP cells were washed with PBS and collected by digestion with 0.25% trypsin without EDTA. Then, NP cells (1 × 10^5^ cells per group) were suspended in 195 μl Annexin V-FITC binding buffer, followed by incubation with 5 μl Annexin V-FITC and 10 μl propidium iodide (PI) for 20 min under dark conditions according to the manufacturer’s instructions (Beyotime, China). Finally, they were subjected to a flow cytometry machine to analyze cell apoptosis ratio. Here, the apoptotic cells including both the early apoptotic cells and the late apoptotic cells are calculated.

### Caspase-3/9 activity measurement

After culture, NP cells were washed with PBS for two times and lysed using 300 μl lysis buffer provided by the test kit (Caspase-3/9 Activity Assay Kit, Beyotime, China) for 10 min. After centrifugation (15,000 rpm, 12 min, 4°C), the supernatant sample was collected and used to perform the chemical reaction according to the method described in the manufacture’s instructions. Finally, their activities were calculated according to the standard curve and the absorbance at a wavelength of 405 nm.

### Real-time PCR analysis

After cultured with different culture medium, NP cells were washed with PBS for two times. Then, total RNA was extracted using TRizol reagent (Invitrogen, U.S.A.) and generated into cDNA using a PrimeScript™ II 1st Strand cDNA Synthesis Kit (TaKaRa, Japan). Gene expression of target genes was analyzed with the method of real-time PCR using an ABI Prism 7700 sequence detection system (Applied Biosystems). The PCR was performed according to the following conditions: 3 min at 95°C, followed by 35 amplification cycles of 10 s at 95°C, 10 s at 55°C, and 10 s at 72°C. Gene primers (Table 1) were synthesized by a bio-company (Sangon Biotech, China). β-actin was used as a reference gene. The method of 2^-△△*C*^_T_ was used to calculate the relative gene expression.

**Table 1:** Primers of target genes

Gene	Forward (5’-3’)	Reverse (5’-3’)
β-actin	CCGCGAGTACAACCTTCTTG	TGACCCATACCCACCATCAC
Bcl-2	GGGGCTACGAGTGGGATACT	GACGGTAGCGACGAGAGAAG
Bax	GGCGAATTGGCGATGAACTG	CCCAGTTGAAGTTGCCGTCT
Caspase 3	GGAGCTTGGAACGCGAAGAA	ACACAAGCCCATTTCAGGGT
Aggrecan	ATGGCATTGAGGACAGCGAA	GCTCGGTCAAAGTCCAGTGT
Collagen II	GCCAGGATGCCCGAAAATTAG	CCAGCCTTCTCGTCAAATCCT
MMP-3	GCTGTTTTTGAAGAATTTGGGTTC	GCACAGGCAGGAGAAAACGA
MMP-13	ATGCAGTCTTTCTTCGGCTTAG	ATGCCATCGTGAAGTCTGGT
ADAMTS-4	ACTGGTGGTGGCAGATGACA	TCACTGTTAGCAGGTAGCGCTTT

### Immunocytochemical staining assay

After culture, NP cells seeded on the glass coverslips were fixed with 4% paraformaldehyde for 20 min. Then, they were permeabilized with 0.1% Triton X-100 for 30 s, blocked with 5% bovine serum albumin (BSA) and incubated with primary antibodies (aggrecan: Novus, NB600-504; collagen II: Abcam, ab185430) overnight at 4°C. After incubation with goat antimouse IgG or goat anti-rabbit IgG (1:400 dilution, Beyotime, China) for 2 h, positive staining was developed and the cellular nucleus was stained with the hematoxylin solution. Finally, staining intensity was analyzed using the Image-Pro Plus software (Version 5.1, Media Cybernetics, Inc.).

### Statistical analysis

Each experiments were performed in triplicate with independent samples. SPSS 17.0 software (Chicago, IL, U.S.A.) was used to analyze the numeric data which were expressed as mean ± standard deviation. The statistical difference was compared using a one-way ANOVA. The *P*-value of 0.05 or less was regarded as a significant difference.

## Results

### Cell apoptosis ratio

Results showed that high glucose culture significantly increased NP cell apoptosis ratio compared with the baseline culture medium. However, the cell apoptosis ratio was partly decreased when OP-1 was added into the high glucose culture medium (Figure 1).

**Figure 1:** Analysis of NP cell apoptosis Data are expressed as mean ± standard deviation, n = 3. *: Indicates a significant difference (*P*<0.05) between two groups.

### Caspase-3/9 activity

Results showed that both caspase-3 activity and caspase-9 activity were significantly increased by the high glucose culture compared with the baseline medium culture. However, their activities were partly decreased by OP-1 addition in a high glucose culture (Figure 2).

**Figure 2:** Analysis of caspase-3/9 activity Data are expressed as mean±SD, n = 3. *: Indicates a significant difference (*P*<0.05) between two groups.

### Gene expression of apoptosis-related molecules

Results showed that high glucose culture significantly decreased gene expression of antiapoptosis molecule (Bcl-2), whereas increased gene expression of pro-apoptosis molecules (Bax and caspase-3) compared with the baseline medium culture. However, their gene expression profiles were partly reversed when OP-1 was added into the high glucose culture medium (Figure 3).

**Figure 3:** Gene expression of apoptosis-related molecules Expression of Bcl-2 mRNA, Bax mRNA, and caspase-3 mRNA was analyzed by real-time PCR. Data are expressed as mean ± standard deviation, n = 3. *: Indicates a significant difference (*P*<0.05) between two groups.

### Gene expression of NP matrix macromolecules

Results showed that gene expression of NP matrix macromolecules (aggrecan and collagen II) was significantly down-regulated in the high glucose culture compared with the baseline medium culture. However, they were up-regulated when OP-1 was added into the high glucose culture medium (Figure 4).

**Figure 4:** Gene expression of NP matrix molecules Expression of aggrecan mRNA and collagen II mRNA was analyzed by real-time PCR. Data are expressed as mean ± standard deviation, n = 3. *: Indicates a significant difference (*P*<0.05) between two groups.

### Gene expression of NP matrix remodeling enzymes

Results showed that gene expression of NP matrix remodeling enzymes (MMP-3, MMP-13, and ADAMTS-4) was significantly up-regulated in the high glucose culture compared with the baseline medium culture. However, all of them were partly down-regulated when OP-1 was added into the high glucose culture medium (Figure 5).

**Figure 5:** Gene expression of NP matrix remodeling molecules Expression of MMP-3 mRNA, MMP-13, and ADAMTS-4 mRNA was analyzed by real-time PCR. Data are expressed as mean ± standard deviation, n = 3. *: Indicates a significant difference (*P*<0.05) between two groups.

### Immunostaining of NP matrix proteins

Results of immunocytochemical staining assay showed that staining intensity of NP matrix proteins (aggrecan and collagen II) was significantly decreased by the high glucose culture compared with the baseline medium culture. However, the staining intensity of them was increased by OP-1 in the high glucose culture medium (Figure 6).

**Figure 6:** Deposition of NP matrix proteins Deposition of aggrecan and collagen II was analyzed by immunocytochemical analysis. Data are expressed as mean ± standard deviation, n = 3. Magnification: 200×, bar = 100 μm. *: Indicates a significant difference (*P*<0.05) between two groups.

## Discussion

Disc degeneration is a main contributor to low back pain. However, its pathogenesis still remains unclear to researchers. Currently, its treatments are just effective to alleviate the pain symptom but not to biologically regenerate/retard disc degeneration. DM is a major public health problem around the world, which has been suggested to be closely related with disc degeneration [9,11,12]. One important reason for disc degeneration in DM patients is that high glucose environment may cause detrimental effects on disc cells through some biochemical signals [10,11,22,23]. Therefore, developing strategies to retarding high glucose environment-induced disc degeneration is important for researchers in the present study field.

The disc contains the central NP, peripheral annulus fibrosus, and cartilage endplate [30]. It has been established that the NP region first exhibits degenerative changes during disc degeneration [31–33]. Hence, we mainly focussed on NP cells in the present study. During disc degeneration, the increased apoptotic NP cells and unbalanced NP matrix metabolism are two important pathological features during disc degeneration [32,34,35]. Here, we confirmed that high glucose microenvironment caused degenerative changes in NP cells and demonstrated for the first time that OP attenuated these degenerative changes in the high glucose culture.

In the present study, we analyzed NP cell apoptosis ratio, caspase-3/9 activity, and gene expression of apoptosis-related molecules (Bcl-2, Bax, and caspase-3) to evaluate NP cell apoptosis. Our results showed that high glucose culture significantly increased cell apoptosis ratio and caspase-3/9 activity, up-regulated expression of pro-apoptosis molecules (Bax and caspase-3), and down-regulated expression of anti-apoptosis molecule (Bcl-2) compared with the baseline culture. These results confirm previous studies that high glucose promotes disc cell apoptosis [18–20]. However, we found that these parameters reflecting NP cell apoptosis exhibited an opposite trend when OP-1 was added into the culture medium in the high glucose culture, indicating that OP-1 may be able to attenuate high glucose environment-induced NP cell apoptosis.

Here, we also observed NP matrix metabolism which was evaluated by gene expression of NP matrix macromolecules (aggrecan and collagen II) and NP matrix remodeling enzymes (MMP-3, MMP-13, and ADAMTS-4), and immuno-staining of NP matrix proteins (aggrecan and collagen II). Results showed that high glucose significantly up-regulated gene expression of MMP-3, MMP-13, and ADAMTS-4, down-regulated gene expression of aggrecan and collagen II, decreased staining intensity of aggrecan and collagen II compared with the baseline culture. These results confirm that high glucose induces matrix catabolism of disc NP cells [10]. Similarly, we found that OP-1 addition partly reversed high glucose-induced NP matrix catabolism, indicating that OP-1 may be able to promote disc NP matrix anabolism in a high glucose microenvironment.

Several limitations of the present study should be noticed. First, the present study is a preliminary study of our research team. Hence, we just focussed on observing cellular changes here, and the possible mechanisms behind this process were not investigated. Previous studies have demonstrated that high glucose environment can induces harmful effects on disc cells through oxidative stress injury [36] or regulating some signaling pathways (i.e., p38 MAPK, PI3K/Akt, and PPARγ-dependent pathway) [20,37,38]. In the future, we will further study the potential mechanism behind the protective effects of OP-1. Second, the rat NP tissue contains many notochordal cells, which will bring some inference to the present results. Third, This is just an *in vitro* study. An *in vivo* animal study should be performed to further verify the protective effects of OP-1 against high glucose-induced degenerative changes of NP cells.

In conclusion, we investigated the effects of OP-1 on high glucose environment-induced degenerative changes in NP cells. Our results demonstrated that OP-1 can alleviate the degenerative changes of NP cells in the high glucose culture. The present study sheds a new light on the strategy to biologically retard disc degeneration in DM patients.

## Abbreviations

ADAMTS: a disintegrin and metalloproteinase with thrombospondin motif-4
Bcl-2: B-cell lymphoma-2
DM: diabetes mellitus
MMP: matrix metalloproteinase
NP: nucleus pulposus
OP-1: osteogenic protein-1
PBS: phosphate buffer solution
